The article "Study on Optimal Extraction and Hypoglycemic Effect of Quercetin" was published in 2023. Journal: Evid Based Complement Alternat Med.

# Study on Optimal Extraction and Hypoglycemic Effect of Quercetin

**DOI:** 10.1155/2023/8886503

**Published:** 2023-08-29

**Authors:** Lei Zhang, Ming-yue Pan, Tao Li, Zhi-min Jin, Zhu Liu, Qiu-yue Liu, Yong Liu, Jia-yuan Ding, Huan Jiang, Xingchen Hou

**Affiliations:** ^1^College of Life Science and Technology, Mudanjiang Normal University, Mudanjiang 157011, China; ^2^Scientific Research Division Sharing Platform for Scientific Research Mudanjiang Medical University, Mudanjiang 157011, China; ^3^Department of Gastroenterology, Hongqi Hospital, Mudanjiang Medical College, Mudanjiang 157011, China; ^4^Jilin University Stomatological Hospital, Jilin 130012, China; ^5^School of Physical Education and Health Sciences, Mudanjiang Normal University, Mudanjiang 157011, China

## Abstract

Quercetin was extracted from *Portulaca oleracea* L. through biphasic acid hydrolysis to investigate its potential as a suppressor of dipeptidyl peptidase IV (DPP-IV) and its hypoglycemic effect in type 2 diabetic mice. The extraction procedure was optimized utilizing the response surface method (RSM) in a single-factor experimental setting. An extraction efficiency of 0.675% was achieved using the following optimized parameters: 0.064 mol/L vitriol, 1 : 109.155 solid-liquid ratio, and 21.408 min ultrasonication. Overall, findings indicate the effectiveness of quercetin extraction. A mouse model for type 2 diabetes was established to receive oral treatment with various quercetin concentrations for 8 weeks. Fasting blood glucose (FBG) and the DPP-IV activity in the serum were significantly reduced. The weight and insulin levels of the mice in the quercetin group were raised compared to those in the model group (*P* < 0.01). Quercetin dose-dependently inhibited postprandial blood glucose excursions, as demonstrated by the oral glucose tolerance test. These results confirmed that quercetin has hypoglycemic effects and considerably improves insulin sensitivity via DPP-IV targeting.

## 1. Introduction

In 2021, according to the most recent data from the International Diabetes Federation, 537 million adults between the ages of 20 and 79 were living with diabetes, accounting for 10.5% of the world's population in this age group. The total number is projected to reach 643 million (11.3% of the world's population) by 2030 and 783 million (12.2%) by 2045 [1]. The most common form of this disease is type 2 diabetes mellitus (T2DM) which amounts to approximately 90% of all cases worldwide. T2DM is recognized as a set of metabolic ailments characterized by hyperglycemia, dyslipidemia, and insulin resistance in target metabolic tissues [2, 3]. Most diabetes' clinical manifestations are characterized by a syndrome of substitution. Some patients have polyuria, polydipsia, increased food intake, and weight loss, as well as an itchy vulva and blurred vision. A prolonged hyperglycemic environment can also result in immune cell abnormalities. These diseases harm multiple organs and result in various common complications. Examples include diabetic cardiomyopathy, diabetic nephropathy, diabetic neuropathy, diabetic wounds, and diabetic retinopathy [4]. Insulin, metformin, sodium-glucose cotransporter 2 (SGLT-2) inhibitors, incretin-based agent-like glucagon-like peptide-1 (GLP-1) receptor agonists (RAs), *α*-glucosidase inhibitors, sulfonylureas (SUF), dipeptidyl peptidase-4 (DPP-4) inhibitors, glinides, and thiazolidinediones (TZDs) are the currently available drugs for the treatment of diabetes [4]. Although the drugs mentioned above are widely used in clinical practice, they can cause side effects.

The article "Study on Optimal Extraction and Hypoglycemic Effect of Quercetin" was published in 2023. Journal: Evid Based Complement Alternat Med.

Traditional herbal remedies have evolved into potentially beneficial biological products that effectively manage or control diabetes. *P. oleracea.* is a medicinal plant that is widely grown in China and is easy to pick, which is rich in flavonoids. Studies have found that flavonoids have obvious hypoglycemic effects [5]. Quercetin is a frequently consumed flavonoid, ubiquitous in beverages and plant-based foods, and abundant in *P. oleracea.* [4, 6]. Like most flavonoids, this pigment typically exists in a range of glycosidic forms rather than as a free aglycone. Most glycosides cannot enter blood due to the obstruction of the small intestine wall; therefore, they must be hydrolyzed into glycosides by hydrolases secreted by probiotics in the intestine and reabsorbed into blood. Only flavones in the form of glycosides can directly enter blood and play various physiological roles. Therefore, quercetin can be detected in plasma after acid hydrolysis. The bioavailability of flavonoid aglycones in vivo is higher than that of flavonoid glycosides [7, 8]. This study aimed to optimize the acid hydrolysis of quercetin from *P. oleracea.* by applying response surface methodology. The treatment was administered to the T2DM mouse model to explore how powerful the hypoglycemic effect is and to understand the underlying mechanisms controlling it.

## 2. Materials and Methods

### 2.1. Experimental Material

Quercetin standards were purchased from Aladdin. Ethanol, hydrochloric acid, and vitriol were acquired from Sinopharm Chemical Reagent Co, Ltd. (Shanghai, China). HPLC-grade methanol was procured from Merck (Darmstadt, Germany). The ICR mice were purchased from Mudanjiang Medical College, and the bioethics protocol number is 20211015-1. *P. oleracea.* was bought from Mudanjiang Pharmacy. High-fat and high-sugar feed was purchased from Xiaoshu Youtai (Beijing) Biotechnology Co., LTD (Table 1). Mouse INS (Insulin) ELISA Kit was bought from Sangon Biotech. STZ was acquired from Beijing DingGuo Biotechnology Company.

The article "Study on Optimal Extraction and Hypoglycemic Effect of Quercetin" was published in 2023. Journal: Evid Based Complement Alternat Med.

### 2.2. HPLC Analysis

The samples were separated into four concentration gradients with concentrations of 0.2 mg/mL, 0.4 mg/mL, 0.8 mg/mL, and 1.0 mg/mL, and the quercetin standard and samples were filtered. As mobile phases for HPLC analysis, methanol (solvent A, 45%) and water (solvent B, 55%) were used at a flow rate of 1 mL/min. The injection volume was 10 *μ*L, the column temperature was 30°C, and the detection wavelength was 360 nm. For linear regression, the peak area of the standard was used as the ordinate, and the mass concentration of the reference product was 1.56, 6.25, 12.5, 25, 50, and 100 *μ*g/mL as the abscissa. The calibration curve is obtained by the formula: *Y* = 11309*X* + 36215 (*R*^2^ = 0.9994).

### 2.3. Extraction of Free and Conjugated Quercetin

Approximately, 900 g of dried and crushed *P. oleracea.* was placed in a 1 L round bottom flask, along with the addition of 80% volume fraction ethanol according to the material-to-liquid ratio of 1 : 7 (m : m), refluxed in a 60°C water bath for 2 h, and extracted for three times in total. All extracts were combined, and the final product was obtained by spinning and steaming under 60°C.

### 2.4. Optimization of Acid Hydrolysis Extraction via RSM

Vitriol and hydrochloric acid were used for these analyses under the following conditions: range of acid concentrations (0, 0.01, 0.05, 0.1, 0.2, 0.4, and 0.8 mol/L), solid-liquid ratios (1 : 10, 1 : 50, 1 : 100, 1 : 150, and 1 : 200), liquid-liquid ratios (1 : 3, 1 : 2, 1 : 1, 2 : 1, and 3 : 1), and extraction times (10, 20, 30, and 40 min). Extraction efficiency was determined based on the observed amounts of extracted target analytes.

To understand the interaction among optimized conditions, RSM was employed by utilizing the Box–Behnken data processor. Based on a single-factor analysis, the quercetin extraction rate was chosen as the dependent variable, whereas solid-liquid ratios, vitriol concentrations, and extraction duration were selected as independent variables. All other conditions were optimized after fixing the extraction temperature at 60°C.

### 2.5. Establishment of the T2DM Mouse Model

Eighty male ICR mice with a weight ranging between 18 and 22 g were exposed to an ambient temperature of 22°C–25°C and a 12 : 12 h light/dark cycle, following housing them in a cage (five animals each). Ten mice in the normal group were given ordinary chow as feed. A high-fat diet was given to the other mice for 1 week. These mice were then made to fast for 8 h; however, they were allowed free access to water. Intraperitoneal injections of STZ (35 mg/kg in 0.1 mol/L citrate-buffered saline, pH 4.4; injection given daily for 3 days) were then given to these mice to induce T2DM. Free access to water and high-fat food were given to the STZ-treated group. The mouse's fasting blood glucose levels were consistently higher than 11.1 mmol/L and remained above 15 mmol/L two hours after gavage, indicating that the model was successfully established.

The article "Study on Optimal Extraction and Hypoglycemic Effect of Quercetin" was published in 2023. Journal: Evid Based Complement Alternat Med.

### 2.6. Treatment Protocol

Five groups of the mice were made, including a quercetin high-dose group that was treated with 80 mg/kg quercetin, a quercetin low-dose group that was treated with 20 mg/kg quercetin, the isoquercitrin group that was treated with 20 mg/kg isoquercitrin, a diabetes model group was treated with 0.9% saline (vehicle), and the normal group was treated with 0.9% saline (vehicle). Among them, sixteen mice were in the high-dose group of quercetin, eighteen mice in the low-dose group of quercetin, eighteen mice in the isoquercetin group, eighteen mice in the diabetes model group, and ten mice in the normal group. Saline (0.9%) was used to dilute all drug stock solutions, administered once daily through oral gavage for 8 weeks. The blood glucose and body weight of mice fasted for 8 h were detected weekly during treatment. Glucose tolerance and serum DPP-IV activity were measured 8 weeks after administration.

### 2.7. Correlation Index Detection

#### 2.7.1. Measurement of Parameters in Serum

Mice were made to fast for 8 h and were tested weekly for DPP-IV during treatment. The suppression effect of serum on DPP-IV was tested in vitro. The tail vein of the mice was used to draw blood samples. The DPP-IV activities were measured by the addition of 10 *μ*L of 10 mmol·L^−1^ Gly-Pro-PNA (the substrate) to a buffer solution (pH 8.0) containing 0.1 mol·L^−1^ NaCl, 1 mmol·L^−1^ ethylenediaminetetraaceticacid (EDTA), 10 mL, and 50 ng DPP-IV and recombinant DPP-IV, respectively, along with or without different concentrations of isoquercetin diluted in dimethylsulfoxide (DMSO). After incubation for 10 min at 37 °C, the reactions were terminated with 0.1 mol·L^−1^ NaHCO_3_, and the amount of the product, pentose nucleic acid (PNA), was measured by UV absorbance at a wavelength of 405 nm. The inhibitory potency of inhibitors was evaluated by IC_50_ values [9]. Based on the GPO-PAP method determined using the instructions in a commercial kit, total cholesterol (TC) and triglycerides (TGs) in serum were calculated. According to the ELISA method, insulin was measured using Mouse INS (Insulin) ELISA Kit.

The article "Study on Optimal Extraction and Hypoglycemic Effect of Quercetin" was published in 2023. Journal: Evid Based Complement Alternat Med.

#### 2.7.2. OGTT Test

After the administration, OGTT tests were performed on mice fasted for 8 hours. Each mouse was given a dose of glucose solution of 2 g/kg by intragastric administration, and glucose content in the caudal vein was measured by using a glucose meter at 0 h, 0.5 h, 1 h, and 2 h, respectively.

### 2.8. Statistical Analysis

Data were presented as the mean ± SD. Using GraphPad Prism 5 software, statistical analysis was conducted using Student's *t*-test or one-way ANOVA. A probability value of *P* < 0.05 was considered statistically significant, and the LSD test was used for postmortem examination.

## 3. Results

### 3.1. Single-Factor Experimental Design

When different solvents were used for extraction, ethyl acetate had a significantly higher extraction efficiency than n-butanol and dichloromethane (Figure 1(a)).

#### 3.1.1. Effect of Vitriol Concentration on Quercetin Extraction

The outcome implies that sulfuric acid is better in terms of its extraction effect than hydrochloric acid. The quercetin extraction rates increased with vitriol concentrations of 0.025–0.1 mol/L but decreased significantly at higher concentrations. The concentration of 0.05 mol/L vitriol was utilized in downstream experiments because peak extraction was achieved at this concentration. It is evident from the observed dose-dependent relationship between extraction efficiency and vitriol concentration that the utilization of high viscosity vitriol solutions may lead to poor penetration of plant raw materials (Figure 1(b)).

#### 3.1.2. Effect of Time on Extraction Efficiency

At extraction times <10 min, the amount of extracted quercetin was low because this timeframe did not furnish sufficient duration to allow solvent penetration into *P. oleracea.* (Figure 1(c)). At extraction times >30 min, the rate of extraction also tends to decline. Peak extraction was observed after 10 min, which was used for subsequent experiments.

#### 3.1.3. Effect of Solid-Liquid Ratios on Quercetin Extraction

A key determinant of extraction efficiency is the ratio of the amount of raw plant material to the amount of solvent. Enhanced extraction efficiency generally results from the high solvent volume; nevertheless, exceedingly large volumes can lead to relatively complex extractions and generate additional unneeded waste.

A notable increase in the quercetin extraction rate was observed when the solid-liquid ratios were maintained between 1 : 50 and 1 : 150 (Figure 1(d)). This finding suggests that the extract was highly viscous at ratios below 1 : 50, thereby resulting in inefficient extraction. An increment in the solid-liquid ratio can result in an enhancement in quercetin extraction. At a ratio of 1 : 100, peak extraction was attained. A 1 : 100 solid-liquid ratio was therefore employed for subsequent single-factor experiments.

The article "Study on Optimal Extraction and Hypoglycemic Effect of Quercetin" was published in 2023. Journal: Evid Based Complement Alternat Med.

### 3.2. RSM-Mediated Parameter Optimization

After the extraction-related parameters were individually evaluated, their interactions were explored via RSM for optimization. These three parameters served as independent variables for this analysis, whereas the dependent variable was taken to be the quercetin extraction index. As detailed in Table 2, experimental randomization was carried out to maximize the influence of inexplicable variability on the extraction rate. Seventeen tests with five replicates (runs 2, 8, 10, 14, and 17, Table 1) were performed to calculate the pure error sum of squares.

The projected *R*^2^ value of 0.7346 corroborated quite well with the adjusted *R*^2^ value of 0.9336. The value of the precision ratio is equivalent to 12.639, suggesting an adequate precision (Table 3). Moreover, the established model had low *P* values (*P* < 0.00001) and extremely high *F* values for a pair of responses. The *F* value of 25.98 indicates only a minimum chance (0.01%) of this value being a consequence of noise. All “Prob > *F*” values of <0.0500 were significant, while values >0.1 were insignificant. Following these specifications, the significant terms in the model are as follows: A, B, C, AB, A^2^, B^2^, and C^2^ (Table 4).

The difference between the predicted *R*^2^ value of 0.7346 and the adjusted *R*^2^ value of 0.9336 was less than 0.2, indicating reasonable agreement. The signal-to-noise ratio is estimated by “Adeq precision.” The desirable ratio is a value greater than 4. The obtained ratio of 12.639 suggests an adequate signal. Hence, the design space can be navigated using this model.

The analysis revealed that the three independent variables were related based on the second-order polynomial expression. Extraction efficiency % = 0.67 + 0.04A + 0.044B + 0.057C + 0.00725AB − 0.00525AC + 0.075BC − 0.38A^2^ − 0.21B^2^ − 0.018C^2^

Figure 2 shows the response surfaces complementing the effect of the independent variables on the mean quercetin extraction efficiency. The interactions between the acid concentration and time, between the acid concentration and solid-liquid ratio, and between the time and solid-liquid ratio are illustrated in Figures 3(a)–3(c), respectively. Predictive software estimated that the extraction efficiency could be as high as 0.675% at a solid-liquid ratio of 1 : 109.155, a vitriol concentration of 0.064 mol/L, and an extraction time of 21.408 min.

### 3.3. Quercetin Reduces Blood Glucose Levels and Ameliorates Body Weight Disorder in T2DM Mice

In T2DM mice, quercetin influences physical characteristics and causes a significant improvement in body weight disorder. When the study began, a T2DM mouse model was created using high-fat feeding and simultaneous low-dose STZ therapy. The outcome suggested the successful creation of the T2DM model: the mice showed polyuria and polydipsia, subsequently losing body weight. The model group exhibited extremely dull hair, high water consumption, and listless spirit compared to the normal group. The quercetin group had a notably better condition than the model group.

The article "Study on Optimal Extraction and Hypoglycemic Effect of Quercetin" was published in 2023. Journal: Evid Based Complement Alternat Med.

Whereas a stable increase in the body weight was observed in the normal mice, a decline was observed in the mouse model (Figure 4(a)). During the early treatment, the value of body weight in the quercetin- and isoquercitrin-treated mice decreased, then underwent a gradual increase, and hardly demonstrated any difference in comparison to that in the normal group. The mice in the quercetin high-dose group and isoquercitrin group showed higher weight than the members of the low-dose group, and the weight shift was more or less dose-dependent. A significant decline was observed in the body weight in the diabetic mouse model following a passage of 8 weeks; however, there was an increase in the other groups of mice. After quercetin and isoquercitrin treatments, the mice's body weight was higher than before treatment (*P* < 0.01). Compared with the normal mice and isoquercitrin-treated mice, the body mass of the quercetin-treated mice manifested no statistically significant difference after therapy. The outcome suggested that quercetin has the potential to ameliorate body weight disorder in T2DM mice. Compared with the model group, the quercetin administration group showed no significant difference in TG and TC contents.

### 3.4. Effect of Quercetin on Glucose Tolerance in Mice

After 8 weeks of mice given quercetin and isoquercetin, the body weight values of mice in the high-dose quercetin group and the isoquercetin group were significantly different from those in the model group (*P* < 0.01), while the low-dose quercetin group was significantly different from the model group (*P* < 0.05) (Figure 4(a)). The blood glucose values of mice in the high-dose quercetin group and the isoquercetin group were very significantly different from those in the model group (*P* < 0.01), while the low-dose quercetin group was significantly different from the model group (*P* < 0.05) (Figure 4(b)). The glucose tolerance values of mice in the high-dose quercetin group and the isoquercetin group were very different from those in the model group (*P* < 0.01), while the low-dose quercetin group was significantly different from the model group (*P* < 0.05) (Figure 4(c)). The increase in the FBG in the diabetic mouse model was relatively gradual and was considerably higher than that in the normal mice (Figure 4(b)). After 8 weeks, the blood glucose level manifested a significant increase in the diabetic mouse model. At the end of the 8-week regimen, the high-dose quercetin group and the isoquercitrin group exhibited a notable decrease in their blood glucose level compared to the diabetic mice (*P* < 0.01). However, there was a noticeable decline in blood glucose levels among the group receiving the low dose (*P* < 0.05). The outcome suggested an efficient hypoglycemic activity of quercetin. Additional *in vivo* investigations, particularly different dosage variants, are key to accurately determining its therapeutic potential. OGTT demonstrated a significant decrease in the blood glucose concentration within the treatment group compared to the model group. Figure 4(c) shows that treatments of isoquercitrin and high-dose quercetin antagonized the blood glucose increase resulting from exogenous glucose and that low-dose quercetin also caused a reduction in the blood glucose level.

The article "Study on Optimal Extraction and Hypoglycemic Effect of Quercetin" was published in 2023. Journal: Evid Based Complement Alternat Med.

### 3.5. Effect of Quercetin Therapy on the Insulin Level and DPP-IV Activity in Serum

In an attempt to address how quercetin exerts its ameliorating effect on hyperglycemia in T2DM mice, the DPP-IV activity in serum was evaluated. There was a rapid decrease in the DPP-IV activity in serum in the diabetic mice that were given quercetin and isoquercitrin treatment. Various quercetin concentrations exhibited a dose-dependent inhibitory impact in the DPP-IV serum of the mice that were treated for 8 weeks (Figure 2(a)).  Figure 2(b) shows that in comparison to those of the model group, the levels of serum insulin of mice in the quercetin group and the isoquercitrin group were considerably higher, in particular in the high-dose isoquercitrin group (*P* < 0.01). The IC_50_ value is 29.6 mg/kg.

## 4. Discussion

Flavonoids are glycosylated derivatives in plant materials, frequently occurring as glycosides [10]. In general, these pigments are absorbed as aglycones after the prior hydrolysis of glycosides along the aerodigestive tract. Hence, the oral flavone glycosides' effect arises from their glycosides' activity [11]. In recent studies, plants containing flavonoids, such as procyanidin, epicatechin, and rhodomyrtone E, have also been indicated to have antiglycation properties [12]. *P. oleracea.* is an annual herb of the family Portulaca oleracea, edible vegetables, and widely planted in the country, has high yield, is easy to pick, and has the effect of reducing swelling and can promote ulcer healing. Quercetin extracted from *P. oleracea.*is less expensive than other hypoglycemic drugs. Quercetin, chemical name 3,3′,4′,5,7-pentahydroxy flavones, is found in many Chinese herbs, mostly in the form of binding glycosides. Acid hydrolysis is a chemical reaction in which an organic molecule is decomposed by water, and acids act as catalysts to hydrolyze glycosides into sugars and aglycones [13]. Quercetin and isoquercitrin are similar in structure and belong to the class flavonoids. Isoquercitrin is hydrolyzed to produce quercetin. In this work, conjugated quercetin was dissociated via acid hydrolysis to increase its extraction rate. The results showed that the extraction rate of quercetin could be improved by adding acids because hydrolysis cleaves the glycoside linkage. Many of the conjugated quercetin molecules are dissociated through acid hydrolysis. Since the dissociation effect of sulfuric acid is enhanced compared to hydrochloric acid, the hydrolysis of flavonoid glycosides proceeded using sulfuric acid as a catalyst [10]. The degradation of flavonoids at high acid concentrations is probably the underlying cause behind the reduction in extraction yields [14]. The continuous extraction of flavonoid glycosides results in a low real-time glycoside concentration, resulting in a noticeable reduction in the required concentration of the acid catalyst. Using a Box–Behnken design, acid hydrolysis was used to determine the optimal conditions for quercetin extraction from *P. oleracea.* The dissociation of conjugated quercetin by acid hydrolysis increased its extraction rate. Vitriol concentration, solid-liquid ratio, temperature and extraction time, and other conditions were optimized for maximal extraction efficiency. RSM with Box–Behnken software was employed to optimize the extraction procedure and explore their associations with one another. For the current analysis, the independent variables were taken as the acid concentration, extraction time, and solid-liquid ratio, whereas the quercetin extraction rate was taken as the dependent variable. The optimized extraction conditions were outlined as vitriol = 0.064 mol/L, ultrasonication time = 21.408 m, and solid-liquid ratio = 1 : 109.155. An extraction efficiency as high as 0.675% could be attained by employing these conditions.

The article "Study on Optimal Extraction and Hypoglycemic Effect of Quercetin" was published in 2023. Journal: Evid Based Complement Alternat Med.

T2DM is characterized by elevated levels of glucose circulating in blood as a consequence of compromised insulin sensitivity of cells (insulin resistance) [15, 16]. The current work revealed important findings about the hypoglycemic influence of quercetin and put forth a novel mechanism, quite independent of preceding works.

Type 2 diabetes and obesity are intricately linked chronic disorders, so the body mass index is a valuable marker for manifesting insulin resistance and glucose tolerance [17]. Quercetin is characterized by alleviation potency on body weight disorder. Oral gavage treatment with various quercetin concentrations led to a profound decrease in hyperglycemia (Figure 4). Glucose tolerance is the embodiment of the body's ability to regulate blood glucose concentration. The high-dose quercetin treatment successfully antagonized the increase in blood glucose caused by exogenous glucose.

Studies have found in mouse models of type 2 diabetes that quercetin regulates hyperglycemia by increasing pancreatic antioxidant levels and enzyme activity associated with glucose metabolism [17]. GLP-1 has been identified as an incretin hormone produced by L cells in the intestine and neurons in the nucleus of the solitary tract (NTS) of the brainstem; together with GLP-1 receptor (GLP-1R), this hormone enhances glycemic control [18–20]. DPP-IV activity is associated with the Glp-1 level in plasma [21, 22] because native GLP-1 undergoes swift degradation by enzyme dipeptidyl peptidase-IV (DPP-IV) [23]. Stable GLP-1 mimetics and DPP-IV inhibitor drugs have been introduced into clinical practice to treat obesity and T2DM [24]. The flavonoid-rich fractions from *Allophylus cominia Sw.* inhibit the DPPIV enzyme [25]. Thus, DPP-IV could be one of the first possible targets of quercetin to improve insulin sensitivity. DPP-IV inhibition may stimulate insulin secretion, which substantially improves the characteristic T2DM symptoms. Zhang et al. [9] reported that quercetin impedes the activity of DPP-IV under in vitro and in vivo conditions, subsequently leading to enhanced secretion of GLP-1 and insulin and ameliorating hyperglycemia in STZ-induced T2DM and high-fat diet mice. Quercetin and isoquercitrin are similar in structure and belong to the class flavonoids. The serum of the mice treated with different quercetin doses showed a significant inhibitory effect on DPP-IV at 8 weeks after administration, and the inhibitory effect increased with the administration dose. Therefore, a reduction in the intensity of hyperglycemia in db/db mice was observed following oral treatment with quercetin. This hypoglycemic potency, in particular, was at least as good as that observed with isoquercitrin. The mechanistic details may point towards improving DPP-IV activity with quercetin; however, this hypothesis requires further studies. In addition, the dose and side effects of quercetin on the human body need to be further studied.

## 5. Conclusion

In conclusion, this study demonstrates that quercetin and isoquercitrin extracted from *P. oleracea.* exert a hypoglycemic effect in a common mouse model of type 2 diabetes. Its function may be related to blood glucose and insulin levels, glucose tolerance, and DPP-IV activity. In addition, it can ameliorate the weight disorder caused by type 2 diabetes. Recent studies [26] and these data support the future use of *P. oleracea.* as a dietary supplement for type 2 diabetes, and it is anticipated that extracted quercetin and isoquercitrin will become new therapeutic agents.

The article "Study on Optimal Extraction and Hypoglycemic Effect of Quercetin" was published in 2023. Journal: Evid Based Complement Alternat Med.

## Figures and Tables

**Figure 1:** Single-factor results: (a) different solvents; (b) sulfuric acid and hydrochloric acid in different concentrations; (c) extraction time; (d) solid-liquid ratio.

**Figure 2:** Effect of quercetin on the insulin level and DPP-IV activity in serum: (a) DPP-IV activity; (b) insulin level. Note: compared with the model group, ^*∗*^*P* *≤* 0.05; ^*∗∗*^*P* *≤* 0.01.

**Figure 3:** Response surface of the effect of factors on quercetin yield.

**Figure 4:** Effect of quercetin on body weight and blood glucose in T2DM mice: (a) effect of drugs on body weight; (b) variation of mouse FBG after treatment; (c) effect of drugs on glucose tolerance.

**Table 1:** List of mouse feed ingredients.

Mouse maintenance feed	High-fat and high-sugar feed
Wheat flour, corn flour, wheat bran,bean cake, dish meal, grass meal	Mouse maintenance feed (66.5%), lard (10%), sucrose (20%), cholesterol (2.5%), sodium cholate (1%)

**Table 2:** Box–Behnken experimental design.

Run	Factor A concentration of vitriol	Factor B extraction time (min)	Factor C solid-liquid ratio (g/mL)
1	0.0625	30	1 : 50
2	0.625	20	1 : 100
3	0.1	20	1 : 150
4	0. 025	10	1 : 100
5	0.1	20	1 : 50
6	0.0625	10	1 : 50
7	0.0625	30	1 : 150
8	0.0625	20	1 : 100
9	0.0625	10	1 : 150
10	0.0625	20	1 : 100
11	0.025	20	1 : 150
12	0.025	20	1; 50
13	0.1	30	1 : 100
14	0.0625	20	1 : 100
15	0.01	10	1 : 100
16	0.025	30	1 : 100
17	0.0625	20	1 : 100

**Table 3:** Credibility analysis of the regression equations.

Index mark	The extraction efficiency of lignans
Std. dev.	0.068
Mean	0.3
C.V. %	22.54
PRESS	0.3
*R*-squared	0.9709
Adj *R*-squared	0.9336
Pred *R*-squared	0.7346
Adeq precision	12.639

**Table 4:** Test of significance for the regression coefficient.

Source	Sum of squares	Df	Mean square	*F* value	*P* value
Model	1.09	9	0.12	25.98	0.0001
A-[BMIM] Br	0.013	1	0.013	2.70	0.1443
B-ultrasonic time	0.016	1	0.016	3.37	0.1092
C-solid-liquid ratio	0.026	1	0.026	5.48	0.0517
AB	0.0002103	1	0.0002103	0.045	0.8382
AC	0.0001103	1	0.0001103	0.024	0.8823
BC	0.022	1	0.022	4.81	0.0644
A^2^	0.60	1	0.60	128.81	<0.0001
B^2^	0.18	1	0.18	38.59	0.0004
C^2^	0.14	1	0.14	30.17	0.0009
Residual	0.033	7	0.004679		
Lack of fit	0.017	3	0.005722	1.47	0.3498
Pure error	0.016	4	0.003897		
Cor total	1.13	16			

The article "Study on Optimal Extraction and Hypoglycemic Effect of Quercetin" was published in 2023. Journal: Evid Based Complement Alternat Med.

## Data Availability

The data used to support the findings of this study are included within the article.
